# Compensated Fuzzy Neural Network-Based Music Teaching Ability Assessment Model

**DOI:** 10.1155/2021/3865190

**Published:** 2021-09-28

**Authors:** Xu Chen

**Affiliations:** College of Teacher Education, Pingdingshan University, Pingdingshan 467000, China

## Abstract

College is the main place to carry out music teaching, and it is important to assess the music teaching ability in college effectively. Based on this, this paper firstly analyzes the necessity of music teaching ability assessment and briefly summarizes the application of neural network and deep learning technology in music teaching ability assessment and secondly designs an assessment model based on compensated fuzzy neural network algorithm and analyzes the accuracy of the model, finds out the causes of forming abnormal output by analysing the general dimensional conditions of the algorithm of the model, and proposes corresponding correction. Finally, the reliability and feasibility of the music teaching ability assessment model were experimentally verified by combining with teaching practice. The research results confirm the feasibility of the compensated fuzzy neural network algorithm in music teaching ability assessment, which has important reference significance for improving the quality of music teaching in colleges and universities.

## 1. Introduction

Music teaching is an important part of the teaching work in colleges and universities, and it is also the main way to improve the music literacy of college students. Compared with conventional teaching methods, diversified music teaching is more relevant and diverse [1]. Colleges and universities not only need to improve students' music literacy in teaching but also need to actively guide students to learn music theory-related knowledge in their daily life [2]. The teaching methods of music teaching include student club activities, music culture festival activities, on-campus music competitions, and classroom lecture teaching. However, the diversity of teaching methods also determines the difficulty of music teaching work in colleges and universities, and how to reasonably evaluate different teaching methods becomes a major difficulty [3]. Low music teaching ability is a common teaching problem in colleges and universities [4]. Music teaching in colleges and universities is currently in a period of transition, and the low teaching efficiency of various teaching methods is an inevitable result [5]. At present, the majority of domestic studies related to the analysis and evaluation of music teaching ability in colleges and universities have been conducted from a developmental perspective, which is not accurate enough and therefore cannot correctly evaluate the level of music teaching in that school [6]. In this context, this paper proposes a music teaching ability assessment model based on compensated fuzzy neural network.

The innovation of this paper is that the research process uses a compensating fuzzy neural network algorithm based on fuzzy decision tree. Compared with the current mainstream research results (evaluation method based on wavelet transform neural network and evaluation method based on dynamic programming strategy), the compensation fuzzy neural network based on particle local learning strategy proposed in this research can conduct in-depth analysis of evaluation model nodes. It solves the short-relevance problem in the traditional music teaching evaluation model and can feedback and evaluate the implementation effect of the evaluation system, and there is no need to consider the time sequence. Based on this, this study uses a fuzzy neural network algorithm to evaluate the music teaching ability of colleges and universities, analyses the existing problems, and greatly improves the evaluation model's evaluation efficiency, accuracy, and reliability of the evaluation results of the music teaching ability of colleges and universities.

The remainder of this paper investigates the influencing factors of music teaching competency assessment and proposes a teaching assessment model based on compensatory neural network, which is divided into four sections.  Section 1 introduces the background of music teaching competency and the general framework arrangement of this section; Section 2 summarizes the current situation of music teaching in colleges and universities and related research on teaching competency assessment and outlines the pain points of current research; in Section 3, we propose a music teaching competency assessment model based on compensated fuzzy neural network; firstly, we give a detailed introduction to overseas research on teaching quality assessment, and then we compare the domestic research, and finally we conclude that the current research on teaching competency assessment lacks a relevant assessment system and assessment model; in Section 4, we take several universities as the experimental objects, obtain the relevant research scales for the study by sampling, and finally, design a music teaching assessment model for universities based on the research scales.

## 2. Related Work

The quality assessment of music teaching in colleges and universities is becoming more and more important [7]. Yadav and Jadhav [8] found that most music teachings in colleges and universities still follow the traditional teaching ideas, ignoring the characteristic indicators and differences of different students' ability to receive music knowledge, so the effect of music teaching in colleges and universities cannot reach the optimal state. Wang and Guo [9] proposed a multistrategy technology-based adaptive model for music teaching assessment in colleges and universities, which solved the problems of inefficiency and low accuracy in the traditional assessment mode. Li [10] analysed students' personality and ability to receive music knowledge to teach different students at different levels of classroom teaching and then realized tiered teaching in the teaching process. Prusa and Khoshgoftaar [11] proved through experiments that the teaching method can well play the role of teaching according to the students' abilities, can effectively improve the effectiveness of music teaching, and used several indicators to assess the students' learning ability. Yang and Zhang [12] found that according to the theory and practical experience of the traditional model of music classroom teaching in colleges and universities, the teaching process in music classroom teaching in colleges and universities pays too much attention to the expression of theory and ignores practice. Parwez et al. [13] proposed an adaptive teaching method based on machine vision algorithm. Smys et al. [14] made students reach a state of deep thinking in the process of learning by conducting listening analysis of different music teaching dialogues and after that experiments proved that the teaching method can well improve the speaking ability in the teaching process of college music teaching classroom and has the advantages of fast teaching speed and obvious effect. Ghosh and Martinsen [15] proposed a new teaching method of college music teaching based on multifactor relationship theory in collaborative science, which analysed the relationship degree of different modules in traditional college music teaching classroom teaching, and established a multifactor coupling analysis model. Bibault et al. [16] conducted a comprehensive evaluation in terms of the choice of teaching format, categorization of teaching content, and students' learning ability using different students for experimental teaching. Alarifi et al. [17] showed that the teaching method of college music teaching based on multirelational recommendation algorithm is better than the classical higher education music teaching pedagogy which is better than the classical higher education music teaching pedagogy. Talasila et al. [18] proposed a tiered teaching method based on music pedagogy theory in order to improve the teaching efficiency and overall stability of higher education music teaching classroom by studying and analysing different students in various aspects. Aminian and Zarenezhad [19] validated it through teaching practice and the final results showed that the teaching method was effective in improving. Forrester [4] proposed a new teaching method for grouped music teaching in colleges and universities based on hyperchaotic mapping, which uses the deformed chaotic sequences to positionally displace the original college music teaching method to achieve an optimal teaching plan for the college music teaching classroom teaching process. Samek et al. [20] have verified the results by practice, and the results show that the teaching scheme of grouped multiple music teaching in colleges and universities has better teaching effect and is suitable for teaching music to junior and senior students.

In summary, it can be seen that most of the current models of teaching music in the college music teaching classroom do not involve intelligent algorithms based on the high and low differentiation of student group characteristics [21]. On the other hand, although a lot of basic research has been done in China on music teaching classroom teaching in colleges and universities, less research has been done on quantitative assessment of music teaching classroom teaching ability in combination with intelligent algorithms [22], and there are also no research and application of unified assessment models for the quality of teaching in music teaching classrooms in colleges and universities in terms of objectivity [23].

## 3. Methodology

### 3.1. Study Population and Study Scale

A total of 60 colleges and universities with music teaching, 30 each of science and technology and comprehensive colleges and universities, which were randomized and volunteered to participate in this study, were selected for the research design of the music teaching evaluation model in colleges and universities under the compensation fuzzy neural network algorithm.  Table 1 shows the general information of the music teaching evaluation model in 60 colleges and universities (polytechnic and comprehensive).

Table 1 shows that the music teaching in the 30 polytechnics is mostly conducted by classroom lectures, accounting for 30/30. 30 comprehensive colleges and universities use independent lectures, accounting for 13/30, and third-party lectures, accounting for 17/30. 30 polytechnics and universities use machine scoring and randomized the music teaching assessment models of the 30 comprehensive colleges and universities which were mostly evaluated manually. In science and engineering colleges and universities, most of the music assessment personnel are counsellors, accounting for more than 90%, while in comprehensive colleges and universities, counsellors and professional music assessment teachers coexist, with counsellors accounting for 40% and professional music assessment teachers accounting for 60%. The number of teachers invested in the process of music teaching assessment in science and engineering colleges and comprehensive colleges is mostly 20∼80 (including the case of one teacher with multiple positions).

There have been many scales for music teaching assessment models in China, such as IPTE (music teaching efficiency), IPTM (music teaching model), IPTD (music teaching orientation), and other scales. In this study, the Generalized Music Teaching Assessment Questionnaire (IPTM-GQ scale) developed by the Institute of Music Education of Renmin University of China is used. The IPTM-GQ scale is the most widely used one, but some practical application effects do not accurately describe the actual situation of music teaching assessment in colleges and universities, so some improvements need to be made to the scale. Specifically, the entries of the IPTM-GQ scale were first translated into Chinese, and the clarity of the expression of the meaning of the items in it was emphasized against other versions of the scale. Considering the excessive differences in the number of items in the IPTM-GQ scale, which is not conducive to the credibility assessment and effect certification degree of this study, we took into account each factor in the process of questionnaire development, consulted relevant information, appropriately screened and added relevant entries, and obtained the following scale, as shown in the first column of Table 2.

In order to reduce the influence of other factors on this study, before the implementation of the revised scale, we need to measure the credibility of the scale and the validity of the effect certification. Thirty colleges and universities of science and technology and comprehensive colleges and universities were selected to conduct the survey. Before the test, the purpose and method of the test were explained to the colleges and universities, and they were required to complete the test within a specified time period. The correlation analysis of each dimension of the scale showed that the correlation data between the effective time of the assessment and other dimensions ranged from 0.58 to 0.94, and the difference dimensions were not significant, indicating that the scale used in this study is suitable for measuring the assessment efficiency of the music teaching assessment model in colleges and universities.

### 3.2. Research Design of Music Teaching Assessment Model in Colleges and Universities under Compensated Fuzzy Neural Network Algorithm

Fuzzy neural network is the product of combining fuzzy theory with neural network, which brings together the advantages of neural network and fuzzy theory and integrates learning, association, recognition, and information processing [24–31]. The fuzzy neural network consists of five layers, which are input layer, fuzzification layer, fuzzy rule layer, fuzzy decision layer, and output layer, and its structure is shown in Figure 1.

In the process of constructing the university music teaching evaluation model based on the compensation fuzzy neural network algorithm, the convolutional neural network constructed includes the input layer, the hidden layer, and the output layer. The input layer can process multidimensional data, and the input layer of a three-dimensional convolutional neural network is used to receive a four-dimensional array. Because convolutional neural networks are widely used in the field of computer vision, this study presupposes three-dimensional input data, that is, two-dimensional pixels and RGB channels on the plane. On the other hand, this study uses the gradient descent algorithm for learning, and the input features of the convolutional neural network need to be standardized. Specifically, before inputting the learning data into the convolutional neural network, the input data need to be normalized in the channel or time/frequency dimension. In addition, the hidden layer of the convolutional neural network includes three common structures: convolutional layer, pooling layer, and fully connected layer. The convolution kernel in the convolutional layer contains weight coefficients, while the pooling layer does not contain weight coefficients. The upstream of the output layer in the convolutional neural network is a fully connected layer, so its structure and working principle are the same as the output layer in the traditional feedforward neural network. For the evaluation of music teaching ability, the output layer uses a logic function or a normalized exponential function to output classification labels. Therefore, the compensation fuzzy neural network algorithm is used to mark the abnormal signals generated in the university music teaching evaluation model and then to carry out the reverse inspection. Discover data information that is different from the signal in the set efficient evaluation state, and then sort out the relevant database information of the marked data information, find the cause of its occurrence, and propose corresponding evaluation suggestions. The preliminary simulation analysis results of the input data are as shown in Figure 2.

As can be seen in Figure 2, the results obtained by the remaining two neural network algorithms show different degrees of perturbative changes compared to the standard dataset, which is due to the fact that compensated fuzzy neural networks have different analysis strategies for different dimensions of data information when processing data. In the research design of the college music teaching evaluation model under this algorithm, the selection of the data processor is crucial and requires us to consider energy consumption, processing speed, and design size. In order to achieve better music teaching evaluation results, the Intel i5 series processor is used in this study. On the other hand, due to the great difference between the devices used, the sensor models collected by different signal ports are different, so this paper designs a suitable working platform according to the different sensor models and divides them into different modules according to the defined configuration of interfaces, interface definitions, wireless communication protocols, etc. This platform is used to collect the data information in the music teaching evaluation model by converting the data information into binary numbers to achieve this; the simulation results of this link are shown in Figure 3.

As can be seen in Figure 3, with the improvement of data information conversion completion under the compensated fuzzy neural network algorithm, the conversion accuracy of all its data information also remained in a high interval range (basically, they all remained around 92%), compared with the remaining two groups of data. In this model of music teaching evaluation based on compensated fuzzy neural network, before analysing the data in the evaluation model, we will set the binary code corresponding to the standard evaluation information, use the compensated fuzzy neural network algorithm to parse the data information in the music teaching evaluation, and compare the binary code of the processed music teaching evaluation information with the standard binary code to filter out the evaluation information that differs from the standard binary code. By backtracking these data, we can indirectly find the root cause of the abnormal data. The abnormal signals of the data were mostly caused by some improper aspects of the music assessment models of the universities, so we organized the data of these abnormal parts and categorized the common information of the abnormal data for nondifferentiated processing, and the simulation results are shown in Figure 4.

As can be seen in Figure 4, under the compensated fuzzy neural network algorithm, there is a significant difference in the error between the two different compensation methods (CFNN1 and CFNN2) compared to the fuzzy neural network (uncompensated FNN), and their convergence values of the error are also different, which is caused by the different focus of the different compensation strategies. In this study, the compensation fuzzy neural network algorithm used to extract the structural type and stability information of the data is mainly divided into two ways: structure learning and parameter learning, and in the process of data learning, the adjustable parameters of different network layers are determined by the parameter learning algorithm, while the determination of the number of neuron nodes in the hidden layer is done according to the structure learning strategy. Therefore, based on this compensation idea, the university music teaching assessment model based on the compensation fuzzy neural network algorithm can be used to find out whether there is abnormal data (improper music assessment module) of low music teaching assessment, mainly based on the following aspects of low assessment efficiency, such as whether the effective time of assessment is less, whether the assessment mode is more traditional, and whether the assessment strategy has not been. The data processing flow is shown in Figure 5.

### 3.3. Mathematical Mechanism Analysis and Simulation Validation of Music Teaching Evaluation Model under Compensated Fuzzy Neural Network Algorithm

In the first step, the secondary validation session of the compensated fuzzy neural network algorithm is performed. We assume that the state variables denote the *s*_*k*_ number of resources allocated from the first detection stage to the final process (*N* stage 1), i.e., the possession of resources associated with the *k* first detection stage; the decision variables *x*_*k*_ denote the allocation of resources in the first stage:

(1) $$\begin{array}{c} S_{k}=\frac{3^{x_{k}}{+4}^{x_{k}}+x_{k}}{2^{x_{k}}+4x_{k}^{2}+5x_{k}^{3}},\\ S_{k+1}=\frac{3^{x_{k+1}}{+4}^{x_{k}}+x_{k+1}}{2^{x_{k+1}}+4x_{k+1}^{2}+5x_{k+1}^{3}}. \end{array}$$

Here, *S*_*k*+1_ with *S*_*k*_ are the expressions in the modified form of

(2) $$\begin{array}{c} S_{k}^{\prime }=\frac{6^{x_{k}}{+5}^{x_{k}}+7x_{k}}{3^{x_{k}}+4x_{k}^{2}+9x_{k}^{3}},\\ S_{k+1}^{\prime }=\frac{5^{x_{k+1}}{+7}^{x_{k}}+7x_{k+1}}{3^{x_{k+1}}+5x_{k+1}^{2}+9x_{k+1}^{3}}, \end{array}$$

where *x*_*k*_ is the decision variable.

The expression for the set of *D*_*k*_(*S*_*k*_) allowed fuzzy decisions without error perturbation analysis *S*_*k*+1_ and *S*_*k*_ is the corresponding set of allowed fuzzy decisions:

(3) $$\begin{array}{c} D_{k}\left(S_{k}\right)=\left\{x_{k}-x_{k-1}|0\leq x_{k}\leq S_{k}\right\},\\ D_{k+1}\left(S_{k+1}\right)=\left\{x_{k+1}-x_{k}|0\leq x_{k+1}\leq S_{k+1}\right\}. \end{array}$$

The expression for the set of *D*_*k*_(*S*_*k*_) allowed fuzzy decisions corresponding *S*_*k*+1_ to the error perturbation analysis *S*_*k*_:

(4) $$\begin{array}{c} D_{k}^{\prime }\left(S_{k}\right)=\left\{\frac{2x_{k}-x_{k-1}}{2x_{k}+x_{k-1}}|0\leq x_{k}\leq S_{k}\right\},\\ D_{k+1}^{\prime }\left(S_{k+1}\right)=\left\{\frac{x_{k+1}-x_{k}}{6x_{k+1}+5x_{k}}|0\leq x_{k+1}\leq S_{k+1}\right\}, \end{array}$$

where *x*_*k*_ is the decision variable in the input layer dataset of the compensated fuzzy neural network.

The optimal indicator functions corresponding to *S*_*k*+1_ and without error perturbation analysis *S*_*k*_ are

(5) $$\begin{array}{c} f_{k}\left(S_{k}\right)=\frac{\text{d}\min_{0\leq x_{k}\leq S_{k}}\left\{g_{k}{\left(x_{k}\right)}^{2}-\sqrt{S_{k+1}}\right\}}{\text{d}x},\\ f_{k+1}\left(S_{k+1}\right)=\frac{\text{d}\min_{0\leq x_{k}\leq S_{k}}\left\{g_{k+1}{\left(x_{k+1}\right)}^{2}-\sqrt{\left(S_{k+2}+S_{k+1}\right)/2}\right\}}{\text{d}x}. \end{array}$$

The optimal indicator functions *S*_*k*_ corresponding *S*_*k*+1_ to the error perturbation analysis are

(6) $$\begin{array}{c} f_{k}^{\prime }\left(S_{k}\right)=\frac{1+\left(\left(\text{d}\min_{0\leq x_{k}\leq S_{k}}\left\{g_{k}{\left(x_{k}\right)}^{2}-\sqrt{S_{k+1}}\right\}\right)/\text{d}x\right)}{2},\\ f_{k+1}^{\prime }\left(S_{k+1}\right)=\frac{1+\left(\left(\text{d}\min_{0\leq x_{k}\leq S_{k}}\left\{g_{k+1}{\left(x_{k+1}\right)}^{2}-\sqrt{\left(S_{k+2}+S_{k+1}\right)/2}\right\}\right)/\text{d}x\right)}{2}, \end{array}$$

where *x*_*k*_ is the decision variable in the input layer dataset of the compensated fuzzy neural network.

Under the compensated fuzzy neural network, *S*_*k*+1_ is the *S*_*k*_ corresponding dynamic programming inverse recurrence relation function:

(7) $$\begin{array}{c} h_{k}\left(S_{k}^{2}\right)=\frac{5S_{k}^{2}+7S_{k}}{k},\\ h_{k+1}\left(S_{k+1}^{2}\right)=\frac{4S_{k+1}^{2}+3S_{k+1}}{k+1}, \end{array}$$

where *x*_*k*_ is the decision variable in the input layer dataset of the compensated fuzzy neural network.

Its combined ground-propagation relation function is

(8) $$\begin{array}{c} h_{k}\left(S\right)=\frac{h_{k+1}\left(S_{k+1}^{2}\right)+h_{k}\left(S_{k}^{2}\right)}{kS_{k+1}^{2}+\left(k-1\right)S_{k}^{2}}. \end{array}$$

In the second step, the weights of the data signals of the tested music teaching assessment models were determined in the analysis process. A total of several groups of experimental tests were carried out, each group had the same initial data information before testing, and the weights of the tested music teaching assessment model in the standard measurement database were 1/5, 1/4, 1/3, 1/2, 1/3, 1/4, and 1/5, and the theoretical measured data results should show a gradually increasing and then gradually decreasing trend.  Figure 6 shows the preliminary simulation analysis results.

As can be seen in Figure 6, the data information recognition rate among the data information gradually becomes larger with the increase of the degree of compensation strategy under the compensation fuzzy neural network algorithm, which is because the data information extraction rules corresponding to different compensation strategies are not the same. The data information recognition efficiency has improved and is within the initial allowable range of this study, which indicates that the compensation fuzzy neural network algorithm has improved the data analysis effect of the college music teaching assessment model and has the condition to detect and analyse the inefficiency of the college music teaching ability assessment model.

In the third step, the database tests the application effect of the college music teaching evaluation model on college music teaching. The host computer used this time is a laptop computer, which is connected to the database of college music teaching assessment of the experimental group and can receive and parse the data packets and store them. By connecting with the signal acquisition end and signal reception end of the college music teaching assessment model, the laptop computer then saves the data stream signals and then parses the data signals to process them, views the expression of the data stream signals with abnormal behaviour, and consults the corresponding college music teaching person in the experimental group if they have similar characteristics when the abnormal signals appear, The head of the teaching assessment model indicated that he or she had similar situations in the daily music teaching assessment process. For example, the effective time of assessment is shorter and the assessment mode is more traditional, which are consistent with the expression of inefficient music teaching assessment. The results of the simulation analysis between assessment efficiency and database data dimensions in this step are shown in Figure 7.

From Figure 7, it can be learned that the measurement efficiency of the three compensation methods (NDN/BPN/CND) gradually decreases with the increase of database dimensionality under the operation of the compensated fuzzy neural network algorithm, which is caused by the fact that the increase of data dimensionality will lead to the increase of computation and the compensation strategy will have been affected to different degrees.

## 4. Current Status of the Efficiency of Music Teaching Assessment in Universities and the Process of Validating the Results

In this study, the current status of the efficiency of music teaching assessment in colleges and universities was detected by using compensated fuzzy neural network algorithm. 60 colleges and universities participated in this experiment, and 49 colleges and universities with low assessment efficiency were detected, with an incidence rate of 81.7%. The feedback survey was conducted on colleges to verify whether the results of this test have high credibility and efficiency certification, and the results show that there are many cases of inefficiency in music teaching assessment in colleges. In addition, the compensation fuzzy neural network teaching ability evaluation model constructed by this research is only applicable to conventional music teaching, such as classical music and pop music, and is not suitable for the evaluation of relatively niche music teaching with local characteristics (for example, ethnic music). The preliminary experimental results of the feedback survey statistics on colleges and universities are shown in Figure 8.

It can be seen from Figure 8 that, in the three groups of experimental data (mixed colleges, polytechnics, and comprehensive colleges), the difference of colleges with assessment efficiency differentiation is more obvious, polytechnics have a high probability of low assessment, which indicates that polytechnics have some problems in music teaching assessment, and compared with comprehensive colleges and mixed colleges, higher vocational colleges still have a certain gap. It should be optimized and adjusted in terms of evaluation mode, evaluation time, and evaluation strategy.

The second step is the validation of the experimental results. In the process of validating the experimental results, we first discuss the relationship between the basic information in the database of music teaching assessment in colleges and universities and the inefficiency of the assessment and analyse the specific reasons.  Table 3 shows the relationship between the management effective time, management mode, management strategy, and scale detection.

From Table 3, we can see that the effective time of evaluation is higher in comprehensive colleges and universities than in polytechnic colleges and universities, and in terms of evaluation mode, polytechnic colleges and universities are significantly higher than comprehensive colleges and universities, and there is no significant difference between polytechnic colleges and comprehensive colleges and universities in terms of evaluation strategy.

## 5. Analysis of Experimental Results

The quantitative assessment of the accuracy analysis of the data obtained in this experiment is shown in Figure 9.

It can be seen from Figure 9 that compared with the current mainstream research results (evaluation method based on wavelet transform neural network and evaluation method based on dynamic programming strategy), the method based on compensated fuzzy neural network proposed in this study gets better evaluation results. In the accurate measurement process of the three evaluation aspects, all showed a gradual increase to a stable process, which shows that the use of the compensation fuzzy neural network algorithm for various data information in the experimental link is still quite high and with the number of iterations. The increase in sigma is gradually in a stable pattern. Therefore, from the above experimental results and analysis process, we can learn that the overall teaching efficiency of music teaching in colleges and universities is low, and the comprehensive colleges and universities are better than the polytechnic colleges and universities, followed by a large difference in effective teaching time, which is caused by the different teaching modes of polytechnic colleges and comprehensive colleges and universities, and from the analysis of colleges and universities themselves, although the teaching mode of polytechnic colleges and universities is based on systematic teaching, which is more from the perspective of colleges and universities, it is relatively efficient and effective in terms of time investment, while the teaching mode of comprehensive colleges and universities is based on “manual + system,” but the effective time of manual teaching is greatly reduced. Although colleges and universities attach great importance to the music teaching assessment model, with the increase of students, the update of the assessment model cannot be synchronized with the actual situation, and the assessment pressure of the music teaching assessment model in colleges and universities has gradually become bigger, and even the situation of music teaching assessment is out of the pit. Therefore, many colleges and universities hope to use lower cost in the process of music teaching assessment, which is also very easy to appear in the situation of low assessment efficiency. Therefore, if we want to further improve music teaching ability and teaching efficiency in colleges and universities, we need to improve from the following aspects:

  First: universities should introduce social resources and use the music teaching experience of social resources to pluck up the music teaching level of universities.
  Second: universities should choose a better assessment teaching mode according to their own advantages. Colleges and universities can set up a college music teaching assessment alliance, build an effective communication platform, and improve the assessment efficiency from many angles.
  Third: colleges and universities should establish an effective music teaching assessment system. Colleges and universities should regularly carry out some activity programs about music teaching for college students to improve their participation in music teaching assessment.

## 6. Conclusion

The traditional music teaching assessment in colleges and universities in China is based on manual assessment, so the efficiency of assessment is very low and the accuracy of assessment is very low. Based on this background, this paper proposes a fuzzy neural network algorithm-based assessment method for music teaching in colleges and universities; firstly, it introduces the current research on the assessment of music teaching ability; secondly, it selects 60 colleges and universities with music teaching courses as the research object and obtains the relevant research quantity through sampling and proposes a new assessment model based on fuzzy neural network; and finally, the new assessment model is used to assess the teaching ability of music teaching in colleges and universities and analyzes the reasons of low efficiency of music teaching in colleges and universities. Finally, the new assessment model is used to evaluate the teaching ability of music teaching in colleges and universities and analyse the reasons for the inefficiency of music teaching in colleges and universities. The experimental results show that the compensated fuzzy neural network algorithm has the evaluation conditions to detect the music teaching evaluation model, can effectively improve the evaluation quality of music teaching in China's colleges and universities, and can normalize the data information in the music teaching evaluation model. Applying the fuzzy control algorithm to the assessment efficiency detection of music assessment in colleges and universities, the rate of low teaching level shown by 30 polytechnic colleges and 30 comprehensive colleges and universities is 81.7%, and the difference of colleges and universities with low teaching ability is more obvious, and the probability of low in polytechnic schools is high, which indicates that polytechnic colleges and universities have some problems in music teaching, compared with comprehensive colleges and universities. Polytechnic colleges and universities should make adjustments in terms of teaching mode, teaching time, and teaching strategies.

## Figures and Tables

**Figure 1:** Compensation of the data processing of the fuzzy neural network algorithm.

**Figure 2:** Simulation data analysis result of compensation fuzzy neural network algorithm.

**Figure 3:** Compensation of the simulation results of the completion and accuracy of data conversion under the fuzzy neural network algorithm.

**Figure 4:** Compensation of the simulation result of the dataset processing amount and error under the fuzzy neural network algorithm.

**Figure 5:** Data processing of music teaching evaluation model.

**Figure 6:** Compensation of the data information extraction rate of different compensation strategies under the fuzzy neural network.

**Figure 7:** Experimental result.

**Figure 8:** Experimental results of compensation fuzzy neural network algorithm.

**Figure 9:** Experimental result.

**Table 1:** General information on the ideological and political teaching management system of 60 colleges (technical and comprehensive).

Category	Science and engineering colleges	Comprehensive colleges
Ideological and political teaching system	Independent research and development	Independent research and development (17/30) + third-party research and development (13/30)
Management approach	System maintenance and random manual maintenance	Manual maintenance
Ideological administrator	Counsellor	Professional ideological construction teacher
Number of teachers	20∼80	20∼80

**Table 2:** Revised IPTM-GQ scale.

	Science and engineering colleges	Comprehensive colleges
Management effective time ratio	0.58	0.61
Management strategy ratio	0.71	0.73
Management mode ratio	0.94	0.88

**Table 3:** Relationship between management effective time, management mode, management strategy, and scale detection.

Ideological and political teaching management system	Management effective time ratio	Management strategy ratio	Management mode ratio
Management effective time ratio	0.98 ± 0.02	0.78 ± 0.01	0.69 ± 0.02
Management strategy ratio	0.77 ± 0.02	0.99 ± 0.01	0.88 ± 0.02
Management mode ratio	0.70 ± 0.02	0.88 ± 0.01	0.98 ± 0.01

## Data Availability

The data used to support the findings of this study are available from the author upon request.
